# The Potential Mechanism of Exercise Combined with Natural Extracts to Prevent and Treat Postmenopausal Osteoporosis

**DOI:** 10.1155/2021/2852661

**Published:** 2021-12-17

**Authors:** Tongxi Zhou, Zhuo Gai, Xing Gao, Li Li

**Affiliations:** College of Sports and Human Sciences, Harbin Sport University, Harbin 150008, Heilongjiang, China

## Abstract

Postmenopausal osteoporosis (PMOP) is a systemic chronic bone metabolic disease caused by the imbalance between bone formation and bone resorption mediated by estrogen deficiency. Both exercise and natural extracts are safe and effective means to prevent and control PMOP. The additive effect of exercise synergy extract against PMOP may be no less than that of traditional medicine. However, the mechanism of action of this method has not been clarified in detail. A large number of studies have shown that the pathogenesis of PMOP mainly involves the OPG-RANKL-RANK system, inflammation, and oxidative stress. Based on the abovementioned approaches, the present study reviews the anti-PMOP effects and mechanisms of exercise and natural extracts. Finally, it aims to explore the possibility of the target of the two combined anti-PMOP through this approach, thereby providing a new perspective for joint intervention research and providing a new direction for the treatment strategy of PMOP.

## 1. Introduction

Postmenopausal osteoporosis (PMOP) refers to women after menopause due to ovarian atrophy, functional degeneration, and estrogen secretion lack, which then induces a reduction in bone mass, bone trabecular structure changes, bone fragility, and easy fracture systemic bone metabolic disease. The traditional prevention method for PMOP mainly uses estradiol and bisphosphonates, but long-term use of such drugs may improve the incidence of cancer and osteonecrosis risk [1]. At present, 200 million women worldwide suffer from osteoporosis. It is expected that by 2050, the number of patients with osteoporotic fractures will double compared with now, which represents a huge medical care and economic burden [2]. Based on this, a proposed study explores the effect of exercise combined with natural extracts on postmenopausal osteoporosis.

## 2. Mechanism of Osteoporosis Formation after Menopause

### 2.1. Bone Resorption Is Uncoupled from Bone Formation

Bone is a multifunctional and changing organ that can support the activities of the motor system and maintain the metabolic balance of minerals such as calcium and phosphate. In order to ensure the homeostasis of the bone microenvironment and meet the needs of body activities, bone tissue should be ablated and regenerated continuously, which is called bone remodeling. Bone remodeling is mainly completed by osteoclasts (OC), osteoblasts (OB), and osteocytes in the bone remodeling cavity. Bone cells in the deep layer of bone can sense the microcracks caused by external force or growth and development, or respond to hormone changes such as estrogen deficiency, transmit signals to the bone surface, and then cause osteoclasts and osteoblasts to function. Osteoclasts are developed from blood-derived mononuclear precursor cells. They are the only bone resorption cells. They can produce enzymes related to the acid dissolution of mineral salts in bone tissue and the degradation of organic matter. They will adhere to the surface of the bone matrix for bone resorption, such as eliminating bone tissue microcracks. In this process, the bone matrix will release a variety of growth factors. Osteoblasts differentiate from bone marrow mesenchymal stem cells and are the main functional cells of bone formation [3]. Stimulated by the direct contact of osteoclasts or cytokines, osteoblasts continue to mature, mineralize, and deposit to form new bone. In this process, osteoblasts can negatively regulate the intensity of osteoclast bone resorption by secreting osteoprotegerin (OPG). Bone remodeling is a dynamic coupling process of bone resorption and bone formation. Therefore, estrogen is very important for the balance of the bone remodeling coupling process.

Both OC and OB are target cells of estrogen, which activates hormone response elements if combined to the estrogen receptor (ER) within OC, can reduce the transcription factor c-jun activity in OC precursors and OC, inhibit osteogenesis induced by RANKL and M-CSF, and attenuate bone resorption [4]. Binding of estrogen to ER also causes upregulation of the apoptosis-associated factor ligand (FASL) of OC that binds to Fas on OC in an autocrine manner and induces OC apoptosis through the Fas/FasL pathway [5]. In OB, estrogen can induce GSK3*β* phosphorylation which blocks *β*-catenin degradation, activates the Wnt/*β*-catenin pathway, binds to the TCF/LEF transcription factor family, and initiates cell cycle genes such as downstream cyc D and c-myc to mediate OB proliferation; and it also upregulates BMP-2 expression, which phosphorylates Smad1/5/8, activates the intranuclear gene expression, and promotes osteogenic differentiation [6]. Estrogen is also able to regulate many transcription factors' activity that in turn inhibits OB apoptosis through activation of Src/Shc/ERK signaling. Less estrogen caused by menopause leads to enhanced OC differentiation and reduced surface FasL expression, and OC escapes apoptosis. It also leads to decreased OB proliferation and differentiation capacity and increased apoptosis. Ultimately, bone resorption capacity is greater than bone formation, causing osteoporosis.

### 2.2. The OPG-RANKL-RANK Signaling System Influences the Bone Remodeling Mechanisms

The OPG-RANKL-RANK signaling system is very important for the process of bone remodeling. Before the discovery of this system, people could not explain the regulatory mechanism of bone resorption and metabolism. Until 1997, Tsuda found a glycoprotein that can specifically inhibit the differentiation of osteoclasts. In the same year, Simonet found a secretory protein that can inhibit the differentiation of osteoclasts and increase bone mineral density. Later, different students found substances with similar functions. After identification, these molecules are the same substance, named osteoprotegerin. The relationship between osteoprotegerin (OPG), nuclear factor-*κ*B receptor activation factor ligand (RANKL), and nuclear factor-*κ*B receptor activation factor (RANK) was found in the subsequent study. In the stable state, the contents of OPG and RANKL are in a balanced state, and their relative contents maintain the number of osteoclasts and support the normal level of bone resorption. When the change of one or more upstream factors excessively tilts this balance to the function of RANKL, the number of active osteoclasts increases and bone resorption is too strong; when the balance tilts too much to the function of OPG, the number of osteoclasts decreases and bone formation is too strong [7].

The mechanisms by which osteoblasts regulate the differentiation and maturation of osteoclasts are influenced by three cytokines, OPG, RANKL, and RANK. RANK belongs to the type I transmembrane receptor protein and is the only receptor for OC surface-mediated RANKL activity, a critical gate for differentiation and activation signaling pathways. RANKL is a member of the tumor necrosis factor (TNF) superfamily that can be secreted by OB, T cells, and endothelial cells and has a role in regulating OC proliferation and differentiation [8].

It has been shown that anti-RANKL treatment can enhance skeletal mechanical properties [9]. Osteoprotegerin, a member of the tumor necrosis factor receptor superfamily, is an osteoclast repressor secreted during OB differentiation and is able to negatively regulate the bone resorption process. OPG acts as an inhibitor of RANK activation by binding to RANKL with a higher affinity, blocking the OC precursor differentiation, inhibiting the function of OC, and preventing excessive bone resorption. Osteoprotegerin presented significant regulation of bone metabolism, with evidence of greater advantage for maintenance of skeletal and muscle function compared to gene deletion or selective inhibition of RANKL, a single treatment with OPG supplementation [10]. Thus, the proportion of OPG/RANKL is the lever that regulates the balance between bone resorption and bone formation. Estrogen downregulates RANKL, induces OC formation, and also promotes OB OPG. The sudden decrease in estrogen secretion after menopause triggered increased RANKL secretion, reduced OPG synthesis, active OC, enhanced bone resorption, and a dynamic imbalance of bone remodeling.

### 2.3. Effects of the Inflammatory Response on Bone Mass

Cells in the bone marrow are functionally divided into cells involved in bone metabolism and hematopoietic cells involved in the immune response, and both share the same microenvironment in the bone marrow and interact to perform functional activities of the skeletal system. It has been clear that osteoclasts and immune cells have common progenitor cells and are also regulated by many common regulators. T cells, B cells, cytokines, chemokines, and costimulatory molecules interact with immune cells under physiological and pathologic conditions, with the OPG-RANKL-RANK signaling system as a bridge to regulate bone formation and bone resorption, and then affect the bone remodeling process [11]. Several studies have shown that almost all chronic diseases are linked to inflammation and that inflammation and immunity are complementary processes, with many immunoactive substances and immune cells involved in the inflammatory response.

B cells and T cells in immune cells are involved in bone formation and bone resorption processes. B lymphocytes were shown to secrete OPG to maintain OPG/RANKL balance and promote bone formation [12]. Interferon *γ* (I FN-*γ*) secreted by helper T lymphocytes 1 (Th1) are important anti-inflammatory factors that have been clinically used in the treatment of severe osteoporosis. IFN-*γ* is able to bind to the OC surface receptor IFNGR, activate TRAFA6, inhibit downstream NF-*κ*B, JNK, and exert antibone resorption; in OB, IFN-*γ* upregulates Runx2, Osterix expression, and osteocalcin and ALP synthesis, which confirmed that the number of OB was significantly decreased in IFN-*γ* receptor gene knockout mice [13]. In contrast to this effect, interleukin 4 (IL-4), mainly secreted by Th2 cells, suppresses OB differentiation by upregulating and downregulating RANKL expression [14]. The specific IL-17 secreted by Th17 in subsets of CD4+ cells can stimulate OB and fibroblasts and also mediate the secretion of the inflammatory factors IL-1, TNF-*α*, and IL-6, further promoting bone resorption and inhibiting bone formation [15]. Furthermore, other inflammatory factors are also involved in the regulation of bone remodeling, and binding of the tumor necrosis factor *α* (TNF-*α*) as a ligand to OC surface receptors can either cooperate with RANKL to induce OC formation or directly activate TRAFA2/6 to upregulate OC expression without RANKL dependence [16]; Smad6/7 activated by TNF-*α* within OB can inhibit Smad1/5/8, to further inhibit BMP-mediated OB differentiation processes. IL-1 is able to bind to OC surface IL1R, which indirectly activates TRAF6, which upregulates OC gene expression through multiple pathways and promotes the bone resorption process [17]. It has also been shown that IL-6 promotes OB-mediated osteogenic differentiation through the activation of JAK 2 and RANKL, and also cooperates with IL-1 and TGF-*β* to induce T cell differentiation into Th17 [18]. There are estrogen targets on T cells that can be directly regulated by the latter, and estrogen can also inhibit the expression of bone resorption factors like TNF-*α*, IL-1, and IL-6 at the gene level, increase the expression of osteogenic factors such as TGF*β*, and then initiate OC apoptosis and prevent bone loss. Submenopausal estrogen reduction leads to T cell expansion, significantly increased content of proinflammatory factors IL-1, IL-6, IL-17, TNF-*α*, and IFN-*γ*, enhanced OC function, reduced OB bone deposition capacity, and bone resorption greater than bone formation, resulting in reduced bone mass and osteoporosis formation [19].

### 2.4. Oxidative Stress Affects Bone Metabolism

Oxidative stress (OS) is also an important pathogenetic factor of postmenopausal osteoporosis. Active oxygen species, such as hydrogen peroxide and hydroxyl groups are produced during cell metabolism, and antioxidant enzyme lines in the body, including catalase (CAT), glutathione catalase (GPX), and superoxide dismutase (SOD), are responsible for removing free radicals from protected cells. Under the dual effects of aging and estrogen reduction, the body's oxidative stress response is enhanced, leading to an imbalance of bone remodeling [20]. In physiological states, intracellular ROS can indirectly activate JNK and serine/threonine kinase (MST1), which then phosphorylates the forkhead transcription factor (FOXO) to nucleate, induce DNA expression, and activate activities like DNA repair, cell cycle, apoptosis, and autophagy [21]. ROS inhibits OB occurrence and reduces its lifespan, so during OB transcription maturation, the transcription factor FOXO protects against increased ROS caused by inducing autophagy and reducing enhanced mitochondrial respiration in osteoblasts [22]. Moreover, FOXO also prevents oxidative stress within OB by increasing SOD, CAT expression, and accumulation of GPX [23]. On the contrary, ROS is required for OC production, function, and survival. ROS can activate JNK and p38 to phosphorylate AP-1 and, in turn, enhance OC differentiation [24], suggesting that FOXO may inhibit bone resorption in an antireactive oxygen species manner. Studies have shown that estrogen can remove reactive oxygen species and protect bone health by fighting body oxidation. Estradiol can significantly enhance autophagy to reduce OB apoptosis through the ERs/ERK/mTOR pathway [25]; RANKL can increase ROS [26], estrogen in osteoclast progenitors can induce the effect of OPG secretion to inhibit RANKL and attenuate the function of OC. Higher serum levels of inflammatory factors and prooxidative biomarkers in menopausal women mean a state of high oxidative stress. Estrogen deficiency increases NADPH oxidase (NOX) on the membrane, decreasing antioxidant system capacity, and ROS accumulation triggers oxidative stress. At the same time, this process exacerbates OB apoptosis and OC differentiation, with bone resorption greater than bone formation and eventually PMOP.

### 2.5. Exercise Affects the Postmenopausal Osteoporosis Mechanism

In recent years, exercise has attracted much attention as a nondrug treatment of osteoporosis. Studies show that exercise effectively controls and prevents osteoporosis and is also a potential intervention strategy to overcome postmenopausal complications due to changes in metabolic hormones, especially estrogen levels [27]. Exercise regulation of the postmenopausal female estrogen secretion mechanism is not clear; the existing studies show the following associations: sports cause the hypothalamus-pituitary-gonadal axis, a study in strict accordance with the ASCM standard for postmenopausal women showed that 12 weeks of exercise can effectively improve female estradiol levels, and compared with aerobic exercise, anaerobic exercise has a more significant effect on bone density [28]. However, the impact of exercise on estrogen secretion is somewhat contradictory. Past studies have shown that adipose tissue can synthesize estrogen, while exercise is conducive to reduce fat quality, so it helps to reduce estrogen levels [29]. Previous studies believe that aerobic exercise has negative effects on estrogen levels, and the effect of resistance exercise is unknown [30]. Another study of postmenopausal obese women showed that estrogen levels increased in aerobic, resistance, and control groups, but there were no significant differences [31]. In short, exercise has a regulatory effect on estrogen, but the specific mechanism and effect results have not been uniformly determined and may be affected by the individual physiological state, exercise strength, and other factors.

A large number of current studies point to the significant positive effect of mechanical loads generated by exercise on maintaining bone mass and that amputation leads to accelerated bone loss in the affected limb [32]. Mechanical stimulation mainly fights the PMOP from several aspects. On the one hand, mechanical load can directly stimulate the ER response and slow down the ER reduction due to estrogen deficiency. Experiments showed that ERK is not activated by pulling tension in OB and osteocytes that knocked down the ER*α* and ER*β* genes, suggesting that ERs are ligand-independent and are directly involved in the conversion of mechanical forces into mechanical signals in osteocytes [33]. On the other hand, mechanical stress may modulate bone remodeling by regulating osteogenic differentiation of myeloid marrow mesenchymal cells. Fluid hydrodynamic regulation of osteogenic differentiation of bone marrow mesenchymal cells is reported to upregulate Runx2 expression in mouse bone marrow mesenchymal cell lines by both classical and nonclassical Wnt pathways, whereas mechanical unloading reduces *β*-catenin expression and suppresses OB proliferation [34]. In addition, exercise also showed upregulation of collagen expression in OB, and mechanical stress affects collagen arrangement upon the formation of new bone, thereby enhancing bone strength. Without physical activity, bed rest or weightlessness negatively affects the bone by inhibiting OB activity and/or enhancing OC activity [35]. In conclusion, the mechanical load induced by exercise has a positive effect on the proliferation and activity of osteoblasts, thereby promoting bone formation under physiological and pathological conditions.

Exercise may cause amelioration of inflammatory cytokines by upregulating anti-inflammatory cytokines, which in turn affect bone metabolism [36]. Low-impact, high-intensity interphase exercise has been reported to stimulate responses to bone transformation markers and cytokines such as IL-1, IL-6, and TNF-*α* which are significantly above baseline, suggesting a correlation between this form of exercise and immune and skeletal responses [37]. The body is in motion. It can also affect the OPG/RANKL/RANK system. Endurance treadmill exercise increases OPG expression and decreases RANKL levels in rats [38]. Resistance exercise increases OPG in adult rats and then upregulates the OPG/RANKL ratio to inhibit bone resorption. Several animal experiments reported similar effects on other forms of exercise: reduced RANKL levels and increased OPG levels were observed in osteoblast experiments in acutely trained mice [39]. Diabetic model rats showed significant OPG in bone and serum and decreased mRNA and protein expression of RANKL after forced swimming training [40]. However, another study found that exercise may not change the level of RANKL and OPG and their expression: a 12-week joint exercise experiment for healthy female college students showed that the bone metabolic response of OPG/RANK/RANKL signaling is not obvious. This speculation is due to the way of exercise. Long-term low-intensity exercise is not enough to improve body function, so the role of the RANKL signaling system is also limited [41]. Long and moderate-intensity regular physical exercise can reduce bone absorption and increase bone mass in healthy people and pathological patients [42]. From the above discussion, it can be concluded that OPG/RANKL changes may be affected by motor mode, motor intensity, and cycle, but still need to be further confirmed by more evidence.

### 2.6. Effects of Natural Plant Extracts on Postmenopausal Osteoporosis

It has been proved that the effective components of various natural plants and Chinese herbal medicines have significant prevention and control effects on PMOP, and the toxic side effects of traditional drug treatment have not been found, which is considered as a potential alternative therapy for traditional drugs for PMOP. It was found that multiple natural components control PMOP as dependent on their estrogen-like effects. It was shown that echinacoside (ECH), a novel phytoestrogen, effectively reverses uterine atrophy in ovariectomy (OVX) rats by enhancing in utero ER expression [43] and upregulating OB proliferation and differentiation via ER-mediated OPG/RANKLER [44]. At the same time, ECH can promote osteogenesis and differentiation of bone marrow mesenchymal cells [45, 46] through activation of the classical Wnt pathway and autophagy; EHC can also regulate the NF-*κ*B pathway and MAPK pathway to inhibit RANKL-induced osteogenesis and reduce bone loss [47]. Similarly, XSPS can promote the nuclear accumulation of *β*-catenin in bone marrow stromal cells without affecting BMP signaling, inducing osteogenic differentiation while inhibiting RANKL induced osteoclast differentiation [48]. Naringin modulates the classical Wnt pathway, upregulates OB differentiation, and downregulates ERK activity, which in turn suppresses bone resorption [49]. Glycyrrhizate directly attenuates OC specific genes and inhibits OC maturation induced by the NF-*κ*B, ERK and MAPK pathways [50]. In addition, genoflavone, soy isoflavone, and resveratrol are also phytoestrogens that can replace estrogen to promote mesenchymal cell osteogenic differentiation and regulate bone remodeling balance [51].

Other native components can also improve bone remodeling imbalance by regulating the OPG/RANKL axis: salidroside  suppresses bone turnover and upregulates bone OPG/RANKL expression, thus increasing bone density in OVX rats [52]. Ginsenoside, the main active ingredient of TCM panax ginseng, significantly suppresses RANKL-induced IKK activity and NFATc1 activity, as well as inhibition of OC synthesis, cathepsin K, MMP, and TRACP, suggesting that ginsenoside can inhibit osteoclast by inhibiting the RANKL-induced NF-*κ*B pathway and Ca^2+^ pathway [53]. Violoxin not only inhibits RANKL mediated expression of OC specific marker genes such as NFATc1 and TRACP, but also promotes expression of factors in OB, thus alleviating bone loss in OVX rats [54]. There is additional evidence that calycosin inhibits the RANKL mediated MAPK pathway and downregulates ALP and TRACP expression [55]. Mountain seed polysaccharide from cypress roots can upregulate OPG to downregulate RANKL expression and regulate the latter-mediated PI3K/Akt pathway [56]. Both components significantly fight osteoporosis in OVX rats, suggesting use as a potential surrogate for PMOP.

Plant components have antioxidative and anti-inflammatory effects, and they realize the prevention of PMOP by preventing inflammation and inhibiting oxidative stress. Epimedii prevents IL-1-induced apoptosis through the PI3K/AKT pathway [57] and also inhibits STAT3 activation and reduces Th-17 cells [58]. Melon polyphenols and lutein are all-natural antioxidants, which have positive effects on protecting bone loss in OVX rats, and lutein can also inhibit OC-specific protein expression and bone resorption [59, 60]. Plant active components can influence oxidative stress levels by upregulating the expression of antioxidant enzyme lines, such as cocoa and lycopene, which can all upregulate GPX and SOD activity within OB and inhibit bone turnover in OVX rats to restore bone strength and microstructure [61, 62]. The advantage of natural ingredients is that there are no toxic side effects. Studies show that pomegranate seed oil extract is rich in phytoestrogens and antioxidants, which have therapeutic effects on osteoporosis and have no adverse effects on blood lipids, uric acid, liver, and kidney function [63]. In conclusion, the estrogen-like effects and antioxidant and anti-inflammatory effects of natural components make them of great research value in the prevention and control of PMOP.

### 2.7. Antimenopausal Osteoporosis Effects of Exercise Combined with Natural Extracts

The PMOP effects of exercise control were limited, and studies showed that exercise intervention in OVX rats could not prevent bone loss after OVX but alleviated the dramatic reduction in estrogen-dependent physiological processes due to estrogen deficiency, and the motor effects were much lower in estradiol than in the OVX rat group [64]. Early studies found that estrogen and mechanical stimulation synergistically inhibit OC generation [65], suggesting that they may work better against PMOP. Alendronate was reported to prevent bone loss in low-intensity whole-body vibration groups in OVX rats, but the combined intervention group was better, suggesting that low-intensity vibration enhances the effect of alendronate on OVX rats by further improving bone trabecular structure [66]. However, high-frequency loading combined with bisphosphonate intervention in OVX rats indicate that a single factor improved bone microstructure, but the combination had no additive effect [67]. The above findings suggest that the effect of the combined intervention may be affected by the exercise mode or exercise intensity as well as the drug type. But traditional drug treatment has limitations and disadvantages, such as estrogen, calcitonin increases the risk of cancer, bisphosphonate has a very low probability of jaw necrosis, and new drugs such as cathepsin K inhibitors, and sclerosing inhibitors clinical application have side effects and lack of long-term efficacy research data [68], which lead to patients' low acceptance and poor compliance with such drug treatments. Natural plant ingredients replace traditional drugs, and in combination with exercise, they may be highly potential and valuable therapies against PMOP.

The effect of PMOP investigated by motion combined with natural extracts is in the exploratory stage, and existing studies illustrate that the efficacy of natural composition and biomechanical stimulation have an additive effect on bone. It is found that the combined intervention can significantly increase the expression of osteoblast transcription factor osterix and inhibit GSK-3*β*, thereby promoting the proliferation and differentiation of osteoblasts and enhancing bone formation. The combination of naringin combined with exercise has been reported to significantly enhance bone strength, bone mass, type I collagen C terminal peptide (CTX), and osteocalcin expression in OVX rats and is superior to a single intervention [69]. The combination of goldfinch isoflavone with resistance exercise prevented femur loss caused by OVX compared to experiments alone [70]. However, the mechanism of joint intervention on PMOP has not been defined, and based on the previous analysis, several pathways of action may involve the following. On the one hand, the estrogen-like effects of natural components can substitute for the mechanical stimulation produced by estrogen synergistic movement and improve bone loss due to hormone deficiency. It has been reported for both phytoestrogen 8-prenylnaringenin (8-PN) and vibration to stimulate ER*α* expression in OVX rats, and it is speculated that vibrations combined with 8-PN stimulation have synergistic effects on OVX rat ER*α*, making the combined group have a more pronounced effect on bone than the 8-PN group [71]. Experiments using rats intervening with the dye lutein (GEN) found a more pronounced reduction in bone mineral density than animals with voluntary exercise. Data show that GEN has no skeletal protection in the absence of physical activity. Meanwhile, the bone-protective effect of GEN may be mediated by ER*α* -dependent mechanisms, and physical exercise has a strong effect on the bone-protective capacity of this phytoestrogen [72]. On the other side, regulation of OPG/RANKL, anti-inflammatory, and antioxidant may also be a combination therapy for anti-PMOP pathway. It was reported that both platform exercise and puerarin alone or combined could downregulate RANKL content in high-fat-raised OVX rats, with no significant effect on mRNA expression of OPG, suggesting that this intervention may be a direct inhibition of RANKL induction of OC formation in OVX rats. Moreover, the combined intervention had a sexual effect on the trabecular quality, and ALP, CTX, and ALP were even better than those of estrogen treatment [73]. A 6-month randomized experiment showed that green tea polyphenols combined with Taijiquan were effective in reducing oxidative stress levels in postmenopausal women, suggesting that the combination therapy may improve PMOP [74]. Through the antioxidant pathway another study showed that soybean isoflavone significantly improved GSH levels in OVX rats but had no SOD activity, while 12-week platform exercise enhanced SOD activity and H_2_O_2_ induced significantly increased DNA tail length, suggesting that moderate exercise binding soy isoflavone protected rats from oxidative stress through different pathways [75]. In addition, isoflavone synergy with weekly aerobic and resistance training for six months reduced TNF-*α* and IL-6 levels in postmenopausal obese women and superior to exercise alone [76].

Furthermore, the combined means may also affect osteogenic differentiation or bone formation marker expression, which in turn affects bone metabolism. It was reported that *β*-catenin, Akt, ER*α*, and Runx2 expression were significantly increased in OB in the treadmill-bound Epimedii intervention group, compared with exercise alone. Combination treatment significantly prevented OVX-induced bone loss and increased OB differentiation and mineralization ability, some of which may be regulated by the ER*α*/Akt/*β*-catenin pathway, but whether combination intervention affected OC differentiation remains unclear [77]. In vitro experiments by domestic scholars have shown icariin combined with exercise coupling stimulation may inhibit bone resorption by regulating NF-*κ*B signaling and influence the upregulation of OB proliferation by the classical Wnt/*β*-catenin pathway. Soybean isoflavone cooperative treadmill exercise intervention can restore bone mass to sham surgical levels in OVX rats with the same effect of estradiol treatment [78]. However, the effect of soy protein combined with moderate endurance exercise in postmenopausal women showed that there was no intervention effect on bone density [79]. In addition, it is speculated that exercise intensity and dosage may affect the combined effect, and the molecular mechanisms of maintaining bone mass may be different, not simply synergy [80].

## 3. Conclusions

In a summary, it is possible that motor binding to natural extracts may involve multiple pathways including mechanical signaling, estrogen deficiency-mediated OPG/RANKL alterations, and anti-inflammatory and antioxidant control of PMOP. Most of the existing studies have shown the additive effect of combination interventions, but several data show no additional efficacy, which may be affected by the choice of exercise regimen and extract dosage. Therefore, the effect and mechanism of combination treatment still need to be further explored by extensive experimental data. Exercise and natural ingredients have great potential and advantages with their low cost, nontoxic, and other advantages, which have been widely valued by the medical community. We are eager to select the best treatment scheme based on various therapies in the future to greatly reduce the pain of patients with osteoporosis and help potential patients stay away from the threat of osteoporosis.

## Data Availability

The data that support the findings of this study are available from the corresponding author upon reasonable request.
